# Hepatic Branch Vagus Nerve Plays a Critical Role in the Recovery of Post-Ischemic Glucose Intolerance and Mediates a Neuroprotective Effect by Hypothalamic Orexin-A

**DOI:** 10.1371/journal.pone.0095433

**Published:** 2014-04-23

**Authors:** Shinichi Harada, Yui Yamazaki, Shuichi Koda, Shogo Tokuyama

**Affiliations:** 1 Department of Clinical Pharmacy, School of Pharmaceutical Sciences, Kobe Gakuin University, Kobe, Japan; 2 Asubio Pharma Co., Ltd., Kobe, Japan; Massachusetts General Hospital/Harvard Medical School, United States of America

## Abstract

Orexin-A (a neuropeptide in the hypothalamus) plays an important role in many physiological functions, including the regulation of glucose metabolism. We have previously found that the development of post-ischemic glucose intolerance is one of the triggers of ischemic neuronal damage, which is suppressed by hypothalamic orexin-A. Other reports have shown that the communication system between brain and peripheral tissues through the autonomic nervous system (sympathetic, parasympathetic and vagus nerve) is important for maintaining glucose and energy metabolism. The aim of this study was to determine the involvement of the hepatic vagus nerve on hypothalamic orexin-A-mediated suppression of post-ischemic glucose intolerance development and ischemic neuronal damage. Male ddY mice were subjected to middle cerebral artery occlusion (MCAO) for 2 h. Intrahypothalamic orexin-A (5 pmol/mouse) administration significantly suppressed the development of post-ischemic glucose intolerance and neuronal damage on day 1 and 3, respectively after MCAO. MCAO-induced decrease of hepatic insulin receptors and increase of hepatic gluconeogenic enzymes on day 1 after was reversed to control levels by orexin-A. This effect was reversed by intramedullary administration of the orexin-1 receptor antagonist, SB334867, or hepatic vagotomy. In the medulla oblongata, orexin-A induced the co-localization of cholin acetyltransferase (cholinergic neuronal marker used for the vagus nerve) with orexin-1 receptor and c-Fos (activated neural cells marker). These results suggest that the hepatic branch vagus nerve projecting from the medulla oblongata plays an important role in the recovery of post-ischemic glucose intolerance and mediates a neuroprotective effect by hypothalamic orexin-A.

## Introduction

Stroke is a devastating disease and a leading cause of death and severe disability worldwide [1]. Risk factors associated with stroke include hypertension, dyslipidemia, and obesity [2], [3]. Additionally, diabetes mellitus and impaired glucose metabolism (e.g. glucose intolerance) are considered to ones of many important risk factors [4]. Past studies have also suggested that hyperglycemia and/or glucose intolerance following stroke may be associated with greater mortality and reduced functional recovery [5], [6]. In a focal cerebral ischemic model, post-ischemic glucose intolerance is one of the triggers of ischemic neuronal damage [7], [8], [9]. However, the mechanisms remain unclear.

Communication between the brain and peripheral tissues, which occurs via the autonomic nervous system, may be essential for maintaining systemic homeostasis, particularly glucose and energy metabolism [10], [11]. In the CNS, the anti-diabetic drug, insulin, suppresses hepatic gluconeogenesis via the hypothalamus and vagus nerve [12], [13]. The hepatic branch vagus nerve provides the primary vagal innervation of the rat liver [14]. Therefore, the precise regulation of liver glucose output is necessary to ensure adequate availability of energy sources for the brain.

The orexin family (orexin-A and orexin-B) are hypothalamic neuropeptides [15] possessing many physiological functions, including arousal and energy metabolism such as glucose metabolism, feeding behavior, sleep and wakefulness [16], [17]. Importantly, orexin-containing axons are widely distributed in the CNS, particularly in areas involved in autonomic regulation [16], [18], [19]. Intra-hypothalamic administration of orexin-A enhances insulin-stimulated glucose uptake by activating the sympathetic nervous system [20]. Furthermore, hyperglycemia in diabetic mice is suppressed by intracerebroventricularly (i.c.v.) administration of orexin-A [21]. In our previous reports, intrahypothalamic administration of orexin-A suppressed cerebral ischemic neuronal damage by regulating post-ischemic glucose intolerance, which was achieved by improving impaired hepatic insulin signaling [8]. In other reports, orexin-positive fibers are shown to be distributed throughout the brainstem, including in neurons of the dorsal motor nucleus of the vagus, which is the major source of parasympathetic innervation to peripheral tissues (such as the liver), and neurons in the nucleus of solitary tract (NTS) [18], [19], [22]. Hence, we hypothesized that regulation of post-ischemic glucose intolerance in subsequent suppression of developed ischemic neuronal damage showed orexin-A in hypothalamus may be mediated to vagus nerves projected from the medulla oblongata to liver.

In the present study, we examined the influence of hepatic branch vagus nerves projected from the medulla oblongata on the recovery of post-ischemic glucose intolerance, and the neuroprotective effect of intrahypothalamic orexin-A administration.

## Materials and Methods

### Animals

The present study was conducted in accordance with the Guiding Principles for the Care and Use of Laboratory Animals, adopted by the Japanese Pharmacological Society. All experimental procedures were approved by the ethical committee for animals at Kobe Gakuin University (approval number: A13-25). Experiments were performed on male ddY mice (5 weeks old, 25–30 g) obtained from SLC (Shizuoka, Japan). Animals were housed between 23–24°C on a 12-hr light–dark cycle (lights on 8:00 a.m. to 8:00 p.m.). Food and water were available *ad libitum*.

### Drug administration in hypothalamus or medulla oblongata

Intra-hypothalamic administration of 5 pmol/mouse orexin-A (Wako, Osaka, Japan), dissolved in saline, was performed immediately after middle cerebral artery occlusion (MCAO). The selective non-peptide orexin-1 receptor antagonist inhibitor, *N*-(2-methyl-6-benzoxazolyl)-*N*′-1,5-naphthyridin-4-yl urea (SB334867) (Tocris Bioscience, St. Louis, MO, USA), was dissolved in 1% DMSO and administered (intramedullary; 50 or 200 pmol/mouse) 30 min before saline or orexin-A intra-hypothalamic administration. The orexin-A and SB334867 doses and the experimental schedule used here were chosen based on our previous publication [8]. All intra-hypothalamic administrations were performed as previously reported [8], [23], [24]. The administration volume for orexin-A and SB334867 was 0.2 µL/mouse. Mice were anesthetized with pentobarbital (40 mg/kg) and immobilized on a stereotaxic instrument (SR-5M; NARISHIGE Co., Ltd., Tokyo, Japan). A microsyringe with a 30-gauge stainless-steel needle was used for all experiments. As previously reported [23], [24] (but with some modifications), the needle was inserted unilaterally into the hypothalamus (1.3 mm posterior to bregma, 0.5 mm lateral from the midline and 5.7 mm deep) and the medulla oblongata (7.8 mm posterior to bregma, 0.5 mm lateral from the midline and 5.2 mm deep). The injection site of the hypothalamus and medulla oblongata was confirmed with 0.5% trypan blue in saline (0.2 µL/mouse).

### Animal model of focal cerebral ischemia

The experimental transient focal ischemia mouse model was induced by performing MCAO, as described previously [25]. Briefly, mice were anesthetized with 2% isoflurane (Abbott Japan, Osaka, Japan) and maintained in an anesthetized state with 1% isoflurane. The common carotid artery (CCA) and external carotid artery were firstly ligated, followed by isolation of the internal carotid artery (ICA). An 8-0 filament (Shirakawa, Fukushima, Japan) coated with a 4-mm thin silicon coat tip (Provil novo Medium; Heraeus Kulzer, Hanau, Germany) was inserted into the left ICA (advanced 9 mm) for 2 h to occlude the left middle cerebral artery (MCA) at its origin through the bifurcation site of CCA. Mice were then anesthetized again, and the occluding filament was gently withdrawn back into the common carotid to allow reperfusion. Sham-operated mice received the same surgery except the filament was not inserted. Body temperature was maintained at 37.0±0.5°C by placing each mouse on a heating pad (FH-100, Unique Medical, Osaka, Japan), which was controlled by a rectal temperature probe (PTE-101, Unique Medical) and a small animal heat controller (ATC-101B, Unique Medical) during surgery and the recovery period. Relative cerebral blood flow (rCBF) was measured by laser Doppler Flowmetry (LDF) (TBF-LN1; Unique Medical) to assess the adequacy of the vascular occlusion and reperfusion, as previously described [25]. MCAO is achieved by a decrease in rCBF to 40% of control values, which is recovered to approximately 100% by reperfusion. In addition, physiological parameters were measured before, during and 30 min after MCAO using a sphygmomanometer (TK-370C; BrainScience Idea, Osaka, Japan) and i-STAT (300F; FUSO Pharmaceutical Industries, Osaka, Japan) [25]. Physiological parameters were within normal physiological ranges in all animals at baseline, during MCAO, and during early reperfusion. We eliminated mice with pricking brain on the silicon coated 8-0 nylon monofilament and unsuccessful infarction on day 3 after MCAO. Thus, the final number of mice was described in each legend. In addition, there are not dead mice by MCAO in present study.

### Measurement of fasting blood glucose (FBG) levels

FBG levels were measured, according to previous reports [8], [26]. Mice were fasted for 15 h and blood samples (∼1.5 µL) were obtained from tail veins. Plasma FBG was measured using the Glucose Pilot (Aventir Biotech, Carlsbad, CA, USA). The increment in FBG was calculated using the following formula: FBG increment  =  FBG on day 1 after MCAO – FBG before MCAO (pre-MCAO FBG), as previously described [26]. The pre-MCAO FBG level was measured at 48 and 96 h before MCAO.

### Measurement of infarct volume

Brains were stained with 2,3,5-triphenyltetrazolium chloride (TTC) (Sigma-Aldrich, St. Louis, MO, USA) to determine infarct volume, as previously demonstrated [8]. Mice were killed on day 3 after reperfusion, and brains were removed, cut (2-mm thick coronal sections) and incubated in saline containing 2% TTC at 37°C for 10 min. Brain slices were then fixed in 4% paraformaldehyde (PFA) at 4°C overnight and scanned. Infarct volumes were measured using the image analysis software, Image J (National Institutes of Health, MD, USA), and Adobe Photoshop Elements 5.0 (Adobe Systems Incorporated, Tokyo, Japan), as previously described [25]. The infarct volume was calculated based on infarct area and intensity (intensity  =  white intensity of left hemisphere – white intensity of right hemisphere) and according to trapezoid formula.

### Neurological examination

Neurological examinations were performed on day 3 after reperfusion using the neurological deficit score (NDS), as previous reported [8], [25]. The NDS consists of consciousness (0, normal; 1, restless; 2, lethargic; 3, stuporous; 4, seizures; and 5, death), walking (0, normal; 1, paw; 2, unbalanced walking; 3, circling; 4, unable to stand; and 5, no movement), limb tone (0, normal; 1, spastic; and 2, flaccid), and the pain reflex. The pain reflex was assessed by the tail flick test (pain reflex  =  latency on day 3 after MCAO – latency before MCAO). NDS points were achieved from the latency difference. A cut-off time of 10 s was used to prevent any injury to the tail. Finally, NDS points assumed total point of consciousness, walking, limb tone and the pain reflex.

### Learning and memory tests

A one-trial step-through-type passive avoidance-learning test was performed to examine learning and memory, as described previously [26]. Briefly, the apparatus (Ohara Co., Ltd., Tokyo, Japan) consisted of illuminated and dark compartments (each 4×13×10 cm) adjoining each other through a small gate (3 cm in diameter) with a grid floor, 2.5 mm stainless steel rods set 7 mm apart. In the training trial (2 days after MCAO), mice were placed in the illuminated compartment facing away from the dark compartment. An electric shock (50 V, 3 s in duration) was delivered when mice entered the dark compartment. They were then returned from the dark compartment to the home cage. In the test trial (on day 3 after MCAO and at 24 h after the training trial), mice were placed in the illuminated compartment, and the latency time to enter the dark compartment (maximum of 600 s) was measured.

### Locomotor activity

Spontaneous locomotor activity was quantified for 30 min by the open field test, as previously described with some modifications [27], [28]. The open field box (30 cm×30 cm×30 cm) consisted of a floor divided into 16 squares (7.5 cm×7.5 cm/square) illuminated by white light. Each mouse was gently placed in the very center of the box and activity was scored as the number of line crossings (i.e. when a mouse removed all four paws from one square and entered another). The open field session was recorded by a camera and the data was analyzed after the session. The open field arena was cleaned with ethanol solution and let dry after testing each mouse.

### Western immunoblot analysis

Western immunoblotting was performed, as described previously [23], [25], [29] but with some modifications. Briefly, the medulla oblongata, liver and skeletal muscle were homogenized in homogenization buffer and diluted with an equal volume of 2× sodium dodecyl sulfate (SDS) sample buffer (0.5 M Tris-HCl [pH 6.8], 10% SDS, 12% β-mercaptoethanol, 20% glycerol, 1% bromophenol blue). Each sample was heated for 3 min at 97°C and protein samples (30 µg) were separated via electrophoresis on 7.5% SDS-polyacrylamide gel and then transferred onto nitrocellulose membranes (BioRad, Hercules, CA, USA) at 15 V for 50 min. Membranes were blocked (60 min at room temperature) in Tris-buffered saline (TBS) (pH 7.6) with 0.1% Tween 20, and either 5% bovine serum albumin (BSA) (Sigma-Aldrich) for insulin receptor (InsR) and tyrosine-phosphorylated (p)-InsR, or 5% skim milk (GE Healthcare, Tokyo, Japan) for orexin-1 receptor, the gluconeogenic regulatory enzymes: phosphoenolpyruvate carboxykinase (PEPCK) and glucose-6-phosphatase (G6Pase), and GAPDH (loading control) (Wako Pure Chemical Industries, Inc., Osaka, Japan). Membranes were incubated with the primary antibodies (in their corresponding blocking solution, overnight at 4°C): rabbit anti-InsR (1∶1000, Abcam, Tokyo, Japan), rabbit anti-p-InsR (1∶500, Abcam), goat anti-orexin-1 receptor (1∶1000, Santa Cruz Biotechnology, Santa Cruz, CA, USA), rabbit anti-PEPCK (1∶1000, Santa Cruz Biotechnology) or goat anti-G6Pase (1∶500, Santa Cruz Biotechnology), and mouse anti-GAPDH (1∶20,000, Chemicon, CA, USA). Blots were then incubated (for 1 h at room temperature) in HRP-conjugated secondary antibodies: anti-rabbit IgG (1∶1,000, KPL, Guildford, UK) for InsR, p-InsR and PEPCK, or anti-goat IgG (1∶1000, KPL) for orexin-1 receptor and G6Pase, and anti-mouse IgG (1∶10,000, KPL) for GAPDH. Immunoreactive bands were visualized with enhanced chemiluminescence western immunoblotting substrate (Pierce; Thermo Scientific, Rockford, IL, USA) followed by a Light-Capture instrument (AE-6981; ATTO, Tokyo, Japan). The signal intensity of immunoreactive bands was analyzed using Cs-Analyzer software (Ver. 3.0) (ATTO) and then normalized to the respective value for GAPDH.

### Immunofluorescence

Immunofluorescence was performed, as described previously [30] but with some modifications. Mice were perfused transcardially with 0.1 M phosphate-buffered saline (PBS) (pH 7.4), followed by 4% PFA in 0.1 M PBS, 9 min after intrahypothalamic administration of orexin-A or saline. The brains (which included the medulla oblongata and hypothalamus) were then cut (2-mm thick slices), and slices were incubated and fixed in ice-cold PBS including 4% PFA at 4°C for 3 h, then dehydrated in 10% followed by 20% sucrose for 3 h followed by overnight, respectively at 4°C. Tissues were then embedded and frozen in the Tissue-Tek optimal cutting temperature compound (Sakura Finetek Japan Co., Ltd., Tokyo, Japan) and stored at −80°C until future use. Frozen blocks were cut into 20 µm-thick sections with a cryostat (Leica CM1850; Microsystems GmbH, Wetzlar, Germany), and mounted on a MAS-coated glass slide (Matsunami Glass Ind., Ltd., Osaka, Japan). Sections were post-fixed in 10% formaldehyde at room temperature for 15 min, and subsequently washed with PBS containing 0.1% Tween 20 (PBS-T) 3 times at 5 min intervals. Sections were exposed to 3% BSA in PBS-T for 1 h at room temperature and then incubated (at 4°C for 48 h) with the primary antibodies (in PBS-T with 1% BSA): goat anti-orexin-1 receptor (1∶100, Santa Cruz) or mouse anti-cholin acetyltransferase (ChAT; 1∶200, Abcam). Sections were incubated (room temperature, 2 h) with the secondary antibody (in 1% BSA): Alexa Fluor 594 goat polyclonal anti-goat (orexin-1 receptor) or -mouse (ChAT) IgG (1∶200, Life Technologies Inc., Carlsbad, CA, USA). Sections were then incubated (in PBS-T with 1% BSA, at 4°C for 24 h) with rabbit anti-c-Fos (1∶2,000, Santa Cruz) for 24 h or ChAT (1∶200) for 48 h. Sections were then washed with PBS-T and incubated (in 1% BSA, at room temperature for 2 h) with the secondary antibody, Alexa Fluor 488 goat polyclonal anti-rabbit (c-Fos) or -mouse (ChAT) IgG (1∶200, Life Technologies). After washing, cover-slips were applied to the sections with Fluoromount/Plus (Thermo Shandon Inc., Pittsburgh, PA, USA). Immunoreactive signals were detected with a confocal laser scanning microscope (FV1000, OLYMPUS, Tokyo, Japan).

### Selective hepatic branch vagotomy

Hepatic branch vagotomy was performed, as described previously [31], [32] but with some modifications. Mice were anesthetized with pentobarbital (65 mg/kg), and the abdominal wall was incised at the midline, the stomach pulled down and the ligaments attaching the liver to the stomach severed. The anterior ligament and the membranous connection of the left lobe of the liver to the diaphragm were cut to provide better visibility of the esophageal-hepatic attachments. The esophageal-hepatic attachment region contains a neurovascular bundle, including the hepatic branch of the vagus nerve. The hepatic branch was selectively transected. Sham vagotomy consisted of the same surgical procedure except for transection of the vagus nerve. MCAO was performed on mice and intrahypothalamic administration of orexin-A or saline was administered on day 7 after surgical recovery.

### Statistical analysis

Infarct volume, FBG and quantification of western immunoblots were analyzed via a one-way ANOVA followed by the Scheffe's test and data are presented by the mean ± SEM. The NDS data and one-trial step-through passive avoidance data were analyzed by the Steel-Dwass test with post-hoc nonparametric multiple comparison tests, and data are presented as medians (25^th^–75^th^ percentile). Significance was reached at values of p<0.05 or p<0.01.

## Results

### Effects of hypothalamic administration of orexin-A on FBG levels and ischemic neuronal damage after MCAO

The injection site of orexin-A in the hypothalamus or SB334867, orexin-1 receptor antagonist, in the medulla oblongata was identified using trypan blue (Figure 1A). Orexin-A significantly suppressed the elevation of FBG levels on day 1 after MCAO compared with the saline-treated group (Figure 2B). Furthermore, orexin-A significantly suppressed the development of infarction, increase of NDS score (neurological abnormalities) and decrease of latency by step-through test (memory disturbances) on day 3 after MCAO compared with the saline-treated group (Figure 1C–F). Administration of SB334867 (200 pmol/mouse) in the medulla oblongata significantly inhibited the effects of orexin-A in the medulla oblongata (Figure 1). SB334867 did not affect body weight, blood glucose levels, food intake, drinking volume, and locomoter activity at 3 days or 7 days after administration of saline (vehicle for orexin-A) or 1% DMSO (vehicle for SB334867) (Figure S1). Expression of orexin-1 receptor was not affected by intrahypothalamic administration of orexin-A (Figure S2).

**Figure 1:** Effects of hypothalamic administration of orexin-A on FBG levels and ischemic neuronal damage after MCAO. Orexin-A (5 pmol/mouse) was intra-hypothalamically administered to mice immediately after MCAO. SB334867 (200 pmol/mouse) was intramedullary administered 30 min before administration of orexin-A. (A) Intra-hypothalamic (upper) or Intra-medullar (lower) administration site (arrow). (B) FBG levels on day 1 after MCAO. (C) Representative photomicrographs of TTC staining on day 3 after MCAO. (D) Quantitative analysis of infarct volume. (B and D) ^**^ *P*<0.01, ^##^ *P*<0.01, ^†^ *P*<0.05. (E) Results of the NDS and (F) the step-through-type passive avoidance learning test on day 3 after MCAO. ^**^ *P*<0.01, ^##^ *P*<0.01, ^†^ *P*<0.05. Sham-treated group: n = 8, MCAO-treated group: n = 6. SAL: saline, OXA: orexin-A.

**Figure 2:** Effects of hypothalamic administration of orexin-A on hepatic and skeletal muscle expression of InsR, p-InsR, PEPCK and G6Pase on day 1 after MCAO. Mice were intrahypothalamically administered with orexin-A immediately after MCAO. SB334867 (50 or 200 pmol/mouse) was intramedullary administered 30 min before orexin-A. Representative western immunoblots and quantification (ratio to GAPDH) as % of sham-SAL of hepatic: InR (A), p-InsR (B), PEPCK (C), G6Pase (D), and skeletal muscular: InsR (E) and p-InsR (F). ^##^ *P*<0.01, ^*^ *P*<0.05, ^#^ *P*<0.05, ^†^ *P*<0.05, Scheffe's test, sham-treated group: n = 6, MCAO-treated group: n = 6. SAL: saline, OXA: orexin-A.

### Effects of hypothalamic administration of orexin-A on hepatic and skeletal muscle expression of InsR, p-InsR, PEPCK and G6Pase after MCAO

Compared with the sham group, protein expression of hepatic InsR and p-InsR was significantly decreased on day 1 after MCAO (Figure 2A, B), which was significantly inhibited by orexin-A (Figure 2A, B). Compared with the sham group, expression of hepatic PEPCK and G6Pase protein was significantly increased in the MCAO group (Figure 2C, D), which was significantly decreased by orexin-A (Figure 2C, D). Similarly, in skeletal muscle, MCAO-mediated decrease of InsR and p-InsR levels on day 1 after MCAO was significantly suppressed by orexin-A (Figure 2E, F). The effects of orexin-A were significantly inhibited by administration of SB334867 (200 pmol/mouse) in the medulla oblongata (Figure 2).

### Co-localization of c-Fos and orexin-1 receptors after intrahypothalamic administration of orexin-A in the medulla oblongata

c-Fos-positive cells were clearly observed in the medulla oblongata (including the NTS) 90 min after intrahypothalamic administration of orexin-A in this region, and was not seen in the sham group (Figure 3A, D). Orexin-1 receptor positive cells were detected in both saline- and orexin-A-treated groups (Figure 3B, E). Furthermore, orexin-1 receptors were co-localized with c-Fos-positive cells in the NTS of medulla oblongata (Figure 3C, F, and Figure S3).

**Figure 3:** Co-localization of c-Fos and orexin-1 receptors after intrahypothalamic administration of orexin-A in the medulla oblongata. Co-localization (C, F) of c-Fos protein (A, D [green]) and orexin-1 receptor (B, E [red]) after saline or orexin-A was intrahypothalamically administered in the medulla oblongata (including nucleus of solitary tract [NTS]). Scale bar: 100 µm. SAL: saline, orexin-1 R: orexin-1 receptor, DMN: dorsal motor nucleus of the vagus.

### Co-localization of c-Fos or orexin-1 receptor with ChAT after intrahypothalamic administration of orexin-A in the medulla oblongata

ChAT-positive cells were detected in the medulla oblongata (including the NTS) in both saline- and orexin-A-treated groups (Figure 4). Furthermore, ChAT-positive cells were co-localized with c-Fos and orexin-1 receptors in the NTS of the medulla oblongata (Figure 4, 5, and Figure S4).

**Figure 4:** Co-localization of c-Fos and choline acetyltransferase (ChAT) after intrahypothalamic administration of orexin-A in the medulla oblongata. Co-localization (C, F) of c-Fos protein (A, D [green]) and choline acetyltransferase (ChAT) (B, E [red]) after intrahypothalamic administration of saline or orexin-A in the medulla oblongata (including the NTS). Scale bar = 100 µm. SAL: saline.

**Figure 5:** Co-localization of ChAT and orexin-1 receptor in naive mice. Co-localization (C, F) of ChAT (A, D [green]) and orein-1 receptor (B, E [red]) after intrahypothalamic administration of saline or orexin-A in the medulla oblongata (including the NTS). Scale bar = 100 µm. SAL: saline, DMN: dorsal motor nucleus of the vagus, 4V: fourth ventricle.

### Effect of hepatic branch vagotomy on orexin-A-mediated suppression of FBG level and neuronal damage after MCAO

The isolation of the hepatic branch of the vagus nerve is shown in Figure 6A. Hepatic branch vagotomy did not affect non-FBG and FBG levels, body weight, food intake, drinking volume, and the expression of InsR, p-InsR, PEPCK and G6Pase in liver or skeletal muscle (Figure S5, S6). Compared with the saline-treated group, hepatic branch vagotomy inhibited orexin-A-mediated suppression of FBG levels on day 1 after MCAO (Figure 6B). In addition, hepatic branch vagotomy inhibited orexin-A-mediated suppression of infarct development, behavioral abnormality and memory disturbance on day 3 after MCAO (Figure 6C–F).

**Figure 6:** Effect of hepatic branch vagotomy on hypothalamic orexin-A-mediated suppression of FBG levels and neuronal damage on day 1 and 3, respectively after MCAO. Intrahypothalamic administration of orexin-A immediately following MCAO on day 7 after hepatic branch vagotomy. (A) Operative field for selective hepatic nerve of the vagus nerve interruption. (B) FBG levels on day 1 after MCAO. (C) Representative photomicrographs of TTC staining on day 3 after MCAO. (D) Quantitative analysis of the infarct volume. (B and D) ^**^ *P*<0.01, ^##^ *P*<0.01, ^*^ *P*<0.05. (E) Results of the NDS and (F) the step-through-type passive avoidance learning test on day 3 after MCAO. ^*^ *P*<0.05, ^#^ *P*<0.05. MCAO/saline-treated group: n = 6, others group: n = 5. SAL: saline, OXA: orexin-A.

### Effect of hepatic branch vagotomy on orexin-A-mediated effects on InsR, p-InsR, PEPCK and G6Pase after MCAO

On day 1 of MCAO, orexin-A restored MCAO-mediated reduction of hepatic and skeletal muscular protein expression of InsR and p-InsR, and the increase of hepatic PEPCK and G6Pase to control levels. This effect was significantly reversed by hepatic branch vagotomy (Figure 7).

**Figure 7:** Effect of hepatic branch vagotomy on hypothalamic orexin-A-mediated effects on hepatic and skeletal muscular expression of InsR, p-InsR, PEPCK and G6Pase on day 1 after MCAO. Intrahypothalamic administration of orexin-A immediately following MCAO 7 days after hepatic branch vagotomy. Representative western immunoblots and quantification (ratio to GAPDH) as % of sham-SAL of hepatic: InR (A), p-InsR (B), PEPCK (C), G6Pase (D), and skeletal muscular: InsR (E) and p-InsR (F). ^*^ *P*<0.05, ^#^ *P*<0.05. n = 12. SAL: saline, OXA: orexin-A.

## Discussion

In recent years, great attention has been given to the regulation of glucose metabolism by not only the control from individual peripheral tissues, such as the liver, but also by the interaction between the hypothalamus and peripheral tissues [10]. Furthermore, the hypothalamus is the most important brain region for the central regulation of glucose homeostasis, where various hormones and neuropeptides cooperate to produce autonomic outflow to the peripheral tissues, such as liver and skeletal muscle [33], [34], [35]. Despite this association, its detailed mechanisms still remain unclear.

We recently reported that the regulation of post-ischemic glucose intolerance by intrahypothalamic administration of orexin-A: (1) restored (to sham levels) the decrease of InsR and the increase of gluconeogenic enzymes in the liver, and (2) significantly suppressed cerebral ischemic neuronal damage [8]. In this study, intrahypothalamic administration of orexin-A significantly increased c-Fos-positive cells in the NTS, which contains the nucleus of the vagus nerve [18]. This result is supported by previous reports demonstrating that i.c.v. administration of orexin-A induces c-Fos activation of NTS neurons [36]. Other reports have shown that orexin fibers are distributed throughout the brainstem, including the dorsal motor nucleus of vague neurons (DMN), which is the major source of parasympathetic innervation to the peripheral tissues (such as the liver) and NTS in the CNS [18], [19]. In addition, orexin-A directly depolarizes the DMN neurons [37]. The NTS (located in the dorsomedial medulla oblongata) is widely accepted to be crucial for the integration of hepatic control mechanisms [38]. Therefore, in the present study, we hypothesized that hypothalamic orexin-A may regulate liver function, such as glucose metabolism, through parasympathetic nerves projected from the medulla oblongata. Thus, we studied the mechanisms underlying the development of ischemic neuronal damage and the role of post-ischemic glucose intolerance, focusing on communication between the brain and peripheral tissues via parasympathetic nerves.

Our findings reveal that the suppressive effect of hypothalamic orexin-A on the development of post-ischemic glucose intolerance and neuronal damage is mediated by orexin-1 receptor in the medulla oblongata. Furthermore, this receptor mediates hepatic InsR and gluconeogenic enzymes after cerebral ischemic stress. These results suggest that hypothalamic orexin-A may affect the liver through the medulla oblongata, specifically the parasympathetic nerve (vagus nerve). Orexin-A has been shown to be densely accumulated in the NTS and DMN, which are involved with efferent parasympathetic nerves and thus more effectively the vagus nerve to the liver [36], [39]. Moreover, orexin-A activates NTS neurons by modulating a nonselective cationic conductance [40], suggesting that orexin-A may have a functional role in the central parasympathetic nerve control of the NTS. Indeed, hypothalamic orexin-A activated NTS and DMN neurons in the medulla oblongata. Furthermore, these activated neurons were co-localized with orexin-1 receptor and ChAT (cholinergic neuronal marker used for the vagus nerve [41], [42]). Therefore, hypothalamic orexin-A-induced effects on liver function (including insulin-induced glucose metabolism) may be mediated by vagus nerves expressing orexin-1 receptor in the NTS of the medulla oblongata. In the hypothalamus, orexin receptors are highly expressed in the LH, the PVN and ARC [43], [44]. These areas are involved in origin of sympathetic or parasympathetic (i.e. the vagus nerve) signals to the liver or skeletal muscle [43], [44]. In our preliminary study, intrahypothalamic orexin-A activated LHA, ARC and PVN-expressing neurons, which were all co-localized with the orexin-1 receptor (data not shown). These results suggest that orexin neurons projecting from the hypothalamus to the medulla oblongata are involved in hypothalamic orexin-A-mediated effects on liver function. However, whether hypothalamic orexin-A affects liver function through the vagus nerve remains unclear. Therefore, this association is under current investigations using hepatic branch vagotomy mice in our group.

Vagus nerve efferents in the common hepatic branch are important for the suppression of hepatic glucose production when the hypothalamic nutrient sensor is stimulated by nutrient repletion signals, such as insulin or fatty acid oxidation [13], [35]. Insulin has been shown over recent years to be a critical determinant of energy homeostasis and peripheral glucose metabolism [45]. Insulin modifies peripheral glucose metabolism (especially liver glucose synthesis) through insulin receptors localized in the hypothalamus [13], [46]. Administration (i.c.v.) of insulin increases insulin sensitivity in peripheral tissues. Furthermore, improved peripheral insulin action is associated with a reduction in hepatic glucose production [13], [46], [47]. The motor nucleus of the vagus mediates hypothalamic insulin signaling via ATP-sensitive potassium (K_ATP_) channels, and reaches the liver via the efferent vagus nerve [13]. Furthermore, activation of either insulin signaling or K_ATP_ channels within the hypothalamus is sufficient to decrease blood glucose levels by a substantial inhibition of glucose production, which is largely due to a marked decrease in the hepatic abundance of gluconeogenic enzymes, such as PEPCK and G6Pase [13], [46], [47]. Also, effects of central insulin and systemic insulin on hepatic glucose production are suppressed [48]. Therefore, activation of the hypothalamus-medulla oblongata-vagus nerve-liver axis is important for insulin signaling on liver function. Changes in glucose uptake in peripheral tissues after intrahypothalamic (VMH) administration of orexin-A have shown that these orexin-A-affected tissues are mediated by the activation of sympathetic nerve signaling with β2-adrenergic receptors in skeletal muscle [20]. Activation of LH and VMH neurons may regulate InsR substrate activity and glucose production in the liver and skeletal muscle via parasympathetic and sympathetic neurons, respectively [49]. That is, it is through that orexin-A is an important to regulate the glucose metabolism in peripheral organs via the activation of the autonomic nervous system. However, the role of endogenous orexin-A in the central regulation of hepatic glucose homeostasis and the vagus nerve (including the hepatic branch vagus nerve) remains to be clarified. Our findings are the first to show that hypothalamic orexin-A affects the vagus nerve-liver axis, and regulates hepatic insulin regulation. More specifically, hypothalamic orexin-A suppressed post-ischemic glucose intolerance by decreasing hepatic InsR and increasing gluconeogenic enzymes via vagus nerve signaling, and also inhibited neuronal damage. In light with these results, other reports have shown that hypothalamic orexin-A levels are significantly decreased by cerebral ischemic stress [8]. These results suggest that the development of post-ischemic glucose intolerance may be involved in the reduction of hypothalamic orexin-A-induced activation of orexin neurons projected from the NTS of the medulla oblongata, causing weakness of vagus nerve stimuli and thus, impairing liver function. However, further study is required to fully elucidate the mechanisms of involvement.

Central actions of insulin are reported to induce the activation of signal transducer and activator of transcription (STAT) 3 phosphorylation in the liver [50], suppresses the expression of the transcriptional coactivator of gluconeogenesis, peroxisome proliferator-acivated receptor γ coactivator-1α, and gluconeogenic genes [50], [51]. Hypothalamic insulin significantly increases both pAkt/Akt and pSTAT3/STAT3 in the liver [52] and thus, may be involved in vagus nerve stimuli projected to the liver [13]. The α7-nicotinic ACh receptor selective agonist, PNU-282987, enhances STAT3 phosphorylation in the liver and skeletal muscle [53]. Hepatic branch vagus nerve leads to the release of ACh, which then binds to muscarinic and nicotinic acetylcholine receptors [54], [55]. Therefore, the regulatory mechanisms of liver function by hypothalamic orexin-A may involve ACh and its receptor, and STAT3. However, this mechanism is still controversial because cholinergic signaling pathways have been reported to not mediate the metabolic effects by the activation of hepatic vagal nerves [56].

However, little is known about the changes in the expression levels of hepatic InsR. Previous reports have shown that polypyrimidine tract-binding protein (PTB) upregulates the expression of insulin and insulin receptor [57], [58]. Under conditions activating insulin signaling, PTB promotes the stabilization of mRNAs encoding insulin and insulin receptor, and enhances the translation of insulin receptor mRNA [57]. Furthermore, CCAAT/enhancer-binding proteins (a family of leucine-zipper transcription factors) regulate the transcription of the InsR as part of a larger nuclear protein complex containing transcription factors such as specific protein 1 [59]. Other reports have demonstrated that TNF-α down-regulates insulin signaling by increasing tyrosine phosphatase 1B [60], suggesting that ischemic stress-mediated increases of inflammatory cytokines may affect the transcription or degradation of the InsR.

In previous finding, orexin-1 receptor, a one of orexin-A receptor, immunoreactivity in the cortex that vulnerable brain region to ischemic stress was increased after cerebral ischemia [61] and i.c.v. orexin-A suppressed the development of infarction through increasing the cerebral blood flow [62]. In addition, in others reports, the mechanisms of the neuroprotective effects of orexin-A have been proved to be related with some intracellular signal transduction pathway, such as hypoxia-inducible factor-1α [63]. That is, these reports suggest that indicated the neuroprotective effect of orexin-A was not only involved in the improvement of post-ischemic glucose intolerance, but also other factors (including other neuroprotective mechanisms such as enhances the cerebral blood flow and inhibits ischemic stress-induced increment of HIF-1α).

In conclusion, these findings provide some insight into the therapeutic effectiveness of this endogenous neuropeptide for its communication between brain and peripheral tissues via the autonomic nervous system, specifically the parasympathetic nerve (vagus nerve).

## Supporting Information

Figure S1 **Changes in body weigh, blood glucose levels, food intake, drinking volume, locomoter activity on day 3 or day 7 after intra-medullar single administration of saline (vehicle of orexin-A) and 1% DMSO (vehicle of SB334867).** (A) Body weight on a daily after administration. (B) Blood glucose levels on a daily after administration. (C) Food intake on day 3 or day 7 after administration. (D) Drinking volume on day 3 or day 7 after administration. (E) Locomoter activity on day 3 after administration. (F) Total count of (E). (F) Locomoter activity on day 7 after administration. (H) Total count of (F). n = 3.
(TIF)

Figure S2 **Effects of hypothalamic orexin-A on changes in orexin-1 receptor on day 1 after MCAO in medulla oblongata.** Mice were intra-hypothalamic administered with orexin-A (5 pmol/mouse) immediately after MCAO. (A) Representative western blots of orexin-1 receptor are shown. (B) Relative levels were analyzed by determining the ratio of orexin-1 receptor/GAPDH on day 1 after MCAO. Results are presented as mean ± S.E.M. n = 4. SAL: saline, OXA: orexin-A.
(TIF)

Figure S3 **Immunohistological expression and co-localization of c-Fos and orexin-1 recepter after intrahypothalamic administration of orexin-A in medulla oblongata.** (A–F) Photomicrographs illustrating the co-localization (C, F) of c-Fos protein (A, D; green) and orexin-1 receptor (B, E; red) after intra-hypothalamic administration of saline or orexin-A (5 pmol/mouse) in medulla oblongata including nucleus of solitary tract (NTS). Scale bar: 100 µm. SAL: saline, orexin-1 R: orexin-1 receptor, DMN: dorsal motor nucleus of the vagus. The dot square showed Figure 3.
(TIF)

Figure S4 **Immunohistological expression and co-localization of c-Fos and choline acetyltransferase after intrahypothalamic administration of orexin-A in medulla oblongata.** (A–F) Photomicrographs illustrating the co-localization (C, F) of c-Fos protein (A, D; green) and choline acetyltransferase (ChAT) (B, E; red) after intra-hypothalamic administration of saline or orexin-A (5 pmol/mouse) in medulla oblongata including nucleus of solitary tract (NTS). Scale bar: 100 µm. SAL: saline. The dot square showed Figure 4.
(TIF)

Figure S5 **Changes in (A) non-fasting blood glucose levels, (B) fasting blood glucose levels, (C) alteration of body weigh (difference of day 7 – day 0), (D) food intake, (E) drinking volume, (F) locomoter activity on day 7 after hepatic branch vagotomy.** n = 3.
(TIF)

Figure S6 **Effect of hepatic branch vagotomy on hepatic and/or skeletal muscular InsR, p-InsR, PEPCK and G6Pase expression on day 7.** Representative western blots of InR, p-InsR, PEPCK, G6Pase and GAPDH levels are shown. Relative levels were analyzed by determining the ratio of InsR/GAPDH, p-InsR/GAPDH PEPCK/GAPDH and G6Pase/GAPDH on day 1 after MCAO. (A) hepatic InsR, (B) hepetic p-InsR, (C) hepatic PEPCK, (D) hepatic G6Pase, (E) skeletal muscular InsR, (F) skeletal muscular p-InsR. Results are presented as mean ± S.E.M. n = 4. SAL: saline, OXA: orexin-A.
(TIF)
